The article "Text Score Analysis under the IPE Environment Based on Improved Transformer" was retracted in 2023. Reasons: unreliable results or conclusions; concerns about the data; concerns about the results or conclusions; concerns about the peer review.

# Text Score Analysis under the IPE Environment Based on Improved Transformer

**DOI:** 10.1155/2022/8354429

**Published:** 2022-09-29

**Authors:** Jinghong Qi, Xinli Jia

**Affiliations:** ^1^Marxism Studies School, Cangzhou Medical College, Cangzhou, 061001 Hebei, China; ^2^Department of Electric Power Engineering, Hebei University of Water Resources and Electric Engineering, Cangzhou, 061001 Hebei, China

## Abstract

In order to improve the accuracy of ideological and political education (IPE) text scoring, an improved short-text similarity calculation model based on transformer is proposed. This model takes the DSSM model as the basic framework and uses the Bert model to realize text representation and solve polysemy problem. The transformer encoding component is used to extract the characteristics of the text and obtain the internal information of the text. With the help of the encoding component, the two texts can interact with information on multiple levels. Finally, the semantic similarity between two texts is calculated by concatenation vector inference.

## 1. Introduction

Natural language processing (NLP) [1] refers to the process of human language into the form of data that can be understood by computers, and the analysis of data and decision-making by simulating the way of thinking of human beings, so as to realize the information exchange between computers and human beings. In today's era of big data, natural language processing technology has become a powerful tool for human to analyze text and mine data. Subjective item is a kind of question which can better test students' knowledge accumulation and subjective cognition. At the same time, it requires the students to reach their own understanding by combining their own knowledge and experience. Teachers need to score students according to their level of literary talent and understanding not just to judge whether they are right or wrong. In recent years, the theory and technology in the field of deep learning are developing vigorously, which strongly promote all walks of life to continuously advance on the intelligent road. Of course, the education industry is no exception, and many intelligent education software have emerged, especially the intelligent demand of homework system and examination system is more and more obvious [2, 3]. At present, due to the unique fixity of the answer itself, the objective question only needs to compare the student's answer with the standard answer to determine whether the question scores or not, so it is a simple programming technical problem. However, the answer to the subjective item is obviously not the only one, and the level of computer intelligence is not comparable to that of the human brain. There is still a certain gap between the scoring effect of the computer to truly achieve the teacher's level, so the automatic scoring technology of subjective item is still difficult to take shape [4]. NLP theory and technology based on deep learning continue to develop and expand, gradually narrowing the gap, making the automatic scoring technology of subjective item get better and better results.

Subjective item is particularly common in the political education classes, relative to other courses, which have stronger subjectivity and flexibility; the score generally has nothing to do with standard answer order of scoring, scoring higher difficulty, so education course subjective item automatic scoring algorithm has the practical value and significance under the background of artificial intelligence and education. First of all, it can help to reduce the score gap caused by the subjective factors of grading teachers and improve the fairness of scoring. Secondly, it can reduce the burden of scientific research workers and teachers on teaching. Finally, it can simplify the whole examination process, improve the efficiency of online education platform, and truly realize intelligent examination [5].

Based on the subjective item of Ideological and political courses, this paper analyzes the characteristics of standard answer text and student answer text. Combined with the deep learning model, the automatic scoring algorithm of subjective item is studied for ideological and political courses. The model takes DSSM model as the basic framework and uses the Bert model to realize the text representation to solve the problem of polysemy.

## 2. Application Status of Short-Text Matching Technology

Short-text matching [6] is a widely used core technology in the field of NLP. It aims to analyze and judge the semantic relationship between two texts. It is widely used in information retrieval [7], question answering system [8], repetition recognition [9], and natural language reasoning [10]. In information retrieval, users want to find documents related to a given query. While for search engines, how to match a given query to the right document is very important. Text matching can also be used to match the right answers for questions in question answering system, which is very helpful for the automatic customer service robot and can greatly reduce the labor cost. Repetition recognition is used to identify whether two natural questions are semantically consistent, while natural language reasoning mainly focuses on whether the hypothetical text can be inferred from the premise text. Therefore, the research on short-text matching is of great significance.

The traditional text matching algorithm mainly solves the problem of word matching at the lexical level, which has some problems such as word meaning limitation, structure limitation, and knowledge limitation. The research on short-text matching has gradually shifted from the traditional statistical method to the deep semantic short-text matching model. In recent years, the pretraining models such as word2vec [11], glove [12], and Elmo [13]. have solved the problem of text vectorization.

At present, most short-text matching models only consider the internal information of text when extracting text features, ignoring the interaction information between two texts, or only carry out single-level interaction, thus losing the rich multilevel interaction information between texts. Information retrieval is also a more complex task, often in the form of Query -- Title, Query -- Document, and a more complex Query might be a Document becoming a Document -- Document, as opposed to other matching tasks. Similarity calculation and retrieval are only a necessary process, more importantly, the need to sort, generally through the retrieval method to recall the relevant items, and then the relevant items rerank. To solve the above problems, we propose an improved short-text matching (ISTM) model based on transformer [14]. ISTM model takes DSSM as the basic framework, uses the Bert model to express the text in vectorization, solves the problem of polysemy of word2vec, and uses the transformer encoder to extract the features of text.

## 3. Text Scoring Model of Ideological and Political Education Based on Improved Transformer

Aiming at the low accuracy of long-text similarity calculation in subjective item, we have transformed the long-text similarity problem into multiple short-text similarity problems in the semantic integrity analysis task. A common solution to this problem is to use keywords to extract feature vectors of long text and then use the similarity between feature vectors to measure the similarity of the corresponding text. The next work is to calculate the short-text similarity, so we propose an improved short-text similarity calculation model based on transformer. The specific implementation steps are as follows:

1. the similarity value between each semantic complete sentence and each score point in the standard answer is calculated by the model
2. then, a score matrix can be obtained by combining the score value of each score point
3. finally, according to certain algorithm, the score matrix selects the score sequence with the highest total score and no overlapping row and column as the final score. Therefore, the process of the algorithm is shown in Figure 1

### 3.1. Transformer Encoder

The transformer encoder has two sub layers, which are multihead self-attention layer and feedforward neural network layer. At the same time, there is a sum layer and normalization step around each sub layer. Its structure is shown in Figure 2, where *N* is the number of encoders.

The dimension of input matrix *X* is *S* × *E*, where *S* is the maximum sequence length, *E* is the dimension of embedding vector, *S* is 25 in this paper, and *E* is 768. The calculation process of the transformer encoder is as follows:

The self-attention mechanism computes query matrix *Q*, key matrix *K*, and value matrix *V* by input matrix *X* and weight matrix *WQ*, *WK*, *WV*, respectively.

(1) $$\begin{array}{c} Q=XW^{Q}, \end{array}$$

(2) $$\begin{array}{c} K=XW^{K}, \end{array}$$

(3) $$\begin{array}{c} V=XW^{V}. \end{array}$$

The output matrix *Z* from the attention layer is calculated

(4) $$\begin{array}{c} Z=\text{Softmax}\left(\frac{QK^{\text{T}}}{\sqrt{d_{k}}}\right)V, \end{array}$$

where *d*_*k*_ is the dimension of the bond vector. *Q* represents the self-attention mechanism computes query matrix; *K* represents the key matrix.

The output matrix *Z*_mul_ of multiple heads from the attention layer is calculated, as shown in Formular (5):

(5) $$\begin{array}{c} Z_{\text{mul}}=\text{Concat}\left(Z_{i}\right)W^{O},i=0,1,\cdots ,H-1, \end{array}$$

where *H* is the number of attention heads, *Z*_*i*_ is the (*i* + 1) attention head, Concat function is the splicing of all *H* attention heads, *W*^*O*^ is the additional weight matrix, and the dimension of *Z*_mul_ is the same as *X*.

Sum and layer normalization are performed, where *LN* function represents layer normalization.

(6) $$\begin{array}{c} Z_{\text{mul}}=LN\left(Z_{\text{mul}}+X\right). \end{array}$$

Finally, *Z*_mul_ is transferred to the feedforward neural network, and then, summation and layer normalization are performed again.

### 3.2. Input of Ideological and Political Text

Text vectorization is an important process in natural language processing. Word2vec is one of the earliest pretraining models. In the past, most of the previous work used word2vec to realize the vectorization of text, which has the advantages of simplicity, high speed, and strong universality. However, it is limited by the corpus. Its modeling is relatively simple and cannot reflect the multilayer characteristics of words, namely, grammar and semantics. Based on transformer, Bert uses the bidirectional encoder structure of transformer, which can reflect the multilayer characteristics of words. This paper uses the Chinese model of BERT-BASE. The model has 12 transformer encoders, each transformer encoder has 12 attention heads, and the hidden layer dimension is 768.

### 3.3. Expression of Ideological and Political Texts

For the multilayer encoder structure of transformer model, it can learn rich syntactic information features in the low-level network, and the higher the level, the closer to semantic information. In order to make the two texts interact in multilevel, we add interactive attention sublayer on the basis of transformer encoder. Suppose that the embedding matrix of the first text is represented *AS* × *E*. The embedding matrix of the second text is expressed as *BS* × *E*. The MP function represents the maximum pooling operation, where *S* is the maximum sequence length and *E* is the dimension of the embedding vector. The output of the two texts after passing through the transformer encoder is as follows:

(7) $$\begin{array}{c} A=\text{Transformer }\left(A\right),\\ B=\text{Transformer }\left(B\right). \end{array}$$

Then, text *A* and text *B* enter the interactive attention sublayer, and the interaction attention moment matrix *M*_S×S_ of the two texts is calculated as follows:

(8) $$\begin{array}{c} \text{M}=\text{A}{\text{B}}^{T}. \end{array}$$

Maximize the pool operation on each line of interactive attention matrix *M* to get vector *r*_*S*_, which represents the attention weight of text B to each character in text *A*. Each element in *r*_*S*_ can be multiplied by each line in *A* to get interactive *A*:

(9) $$\begin{array}{c} \text{A}={\text{MP}}_{\text{row}}\left(\text{M}\right)\times \text{A} \end{array}$$

Maximize the pooling of each column of the interactive attention matrix *M* to obtain vector *c*_*S*_, which represents the attention weight of text *A* to each character in text *B*. The interactive *B* can be obtained by multiplying each element in *c*_*S*_ by each line in *B*:

(10) $$\begin{array}{c} \text{B}={\left[{\text{MP}}_{col}\left(\text{M}\right)\right]}^{T}\times \text{B} \end{array}$$

In this way, each time the two texts are encoded, they will have an information exchange. According to the number of encoders, the two texts can interact with each other at different levels, which can not only encode the context information in depth but also obtain the enhanced interactive information.

### 3.4. Similarity Prediction of Ideological and Political Texts

After passing through the presentation layer, the two texts are encoded as matrix tables with rich contextual and interactive information, assuming *A*_*S*×*E*_ and *B*_*S*×*E*_, respectively. At the prediction layer, matrix *A* and matrix *B* are maximized and the vectors of two texts are divided to represent *v*_*A*_ and *v*_*B*_. Then, the similarity between the two texts can be calculated as follows:

(11) $$\begin{array}{c} y^{\prime }=F\left(\left[{\text{v}}_{A};{\text{v}}_{B};{\text{v}}_{A}\times {\text{v}}_{B};\left|{\text{v}}_{A}-{\text{v}}_{B}\right|\right]\right). \end{array}$$

Among them, the *y*′ indicates the similarity prediction between two texts, |*v*_*A*_ − *v*_*B*_| emphasizes the difference between two texts, *F* function means that the splicing vectors of the four vectors are input into the fully connected neural network, and then, the predicted value of the output text similarity is calculated by sigmoid function. In addition, if the sigmoid function is replaced by the Softmax function, the model can be used as a short-text matching model to deduce the semantic relationship between two texts for short-text matching tasks.

### 3.5. Score Calculation

Through the short-text similarity calculation model, we can calculate the similarity value between each score point in the standard answer and each semantically complete sentence in the student answer, and then combining the score value of each score point, we can get a score matrix *S*_*N*×*M*_, where *N* is the number of score points and *M* is the number of semantically complete sentences. Suppose the matrix representing the set of points is {*P*_0_, *P*_1_, ⋯, *P*_*N*−1_}, the matrix of student's answer clause represents the set {*A*_0_, *A*_1_, ⋯, *A*_*M*−1_}; STS function represents the short-text similarity calculation model; then, the calculation formula of each element in the score matrix is as follows:

(12) $$\begin{array}{c} s_{ij}=\text{STS}\left(P_{i},A_{j}\right),i=0,1,\cdots ,N-1,j=0,1,\cdots ,M-1 \end{array}$$

The next work is to select the score according to the score matrix to calculate the final score of students' answers. It should be noted that every time a score is selected, the peer or column elements of the score cannot be selected, because it is necessary to ensure that a score point in the final score sequence corresponds to a student's answer clause. Otherwise, it may lead to a student's answer clause scoring at multiple scoring points.

## 4. Experiment and Analysis

### 4.1. Data Set

The automatic scoring algorithm of subjective item is studied for ideological and political courses. For the task of semantic integrity analysis, we collected Ma Yuan, Mao Gai, and Si Xiu's modern history and other ideological and political corpus. After removing redundant and useless characters from the original corpus, we got 12400 semantic complete sentences, about one million characters. Then, the order of the sentences is disrupted to make the data more evenly distributed, and each character is marked by Jieba part of speech tagging combined with manual tagging, and the sentences are separated by a new line. Finally, the data set was segmented in a ratio of 6 : 2 : 2.

Due to the scarcity of Chinese subjective item scoring data sets, we collected a certain number of “standard answer-student answer” answer data sets based on ideological and political course exams, among which each course accounted for a relatively balanced proportion. 1000 score-student answer clauses were extracted from these answer pairs, and the similarity value was marked to each sentence pair according to their ratio, so as to obtain the data set of short-text similarity calculation task. We also segmented the data set according to the ratio of 6 : 2 : 2. In addition, we retained 100 answer pairs and scaled the total score to 10 points for the automatic scoring of the whole subjective item.

### 4.2. Model Parameters

The main model parameters set in this experiment are shown in Table 1.

When training the model, we need to pay attention to the convergence of the model. If the model converges, we should stop training; otherwise, the model will overfit and fail to achieve the desired effect. The convergence of short-text matching model is shown in Figure 3.

As shown in Figure 3, the model has begun to converge after the training times exceed 25, so set the training times to 30.

### 4.3. Evaluation Index

Recall and precision are the best tools to measure the accuracy of prediction model. The model in this paper also uses these two concepts to judge. By constantly adjusting the sampling mode and proportion, the accuracy of the model is constantly improved. We use F1 value and accuracy Acc as indexes to evaluate the model, with *F* value as the main factor and accuracy rate as the auxiliary. The value of *F* is obtained from *P* and *R*, and the relevant calculation formula is as follows:

(13) $$\begin{array}{c} P=\frac{TP}{TP+FP} \end{array}$$

(14) $$\begin{array}{c} R=\frac{TP}{TP+FN} \end{array}$$

(15) $$\begin{array}{c} F1=\frac{2\times P\times R}{P+R} \end{array}$$

(16) $$\begin{array}{c} Acc=\frac{TP+TN}{TP+TN+FP+FN} \end{array}$$

where TP represents the positive case when the actual result is positive, FN represents the negative case when the actual result is positive, FP represents the positive case when the actual result is the negative example, and TN represents the counter example when the actual result is the counter example.

### 4.4. Results and Discussion

#### 4.4.1. Comparison Results of Different Models

Several classic text matching models are selected for experimental comparison. RNN (Experiment 1), BIRNN (Experiment 2), GRU (Experiment 3), BiGRU (Experiment 4), LSTM (Experiment 5), and BiLSTM (Experiment 6) were added as comparative experiments. In addition, in order to enhance the parallel computing ability and feature extraction ability, Zhao proposed to replace the deep neural network of DSSM with transformer coding component. Therefore, in order to enhance the contrast effect, transformer DSSM (Experiment 7) [15] is also used in comparative experiments. Moreover, Experiment 8 represents our models.

The experimental results of each model are shown in Figure 4, where the abscissa is the experimental number, and the ordinate is the percentage value of different indexes. The text vectorization mode adopted by the model is BERT by default; otherwise, it is Word2vec.

The results show that the F1 value of the LSTM model can reach 86.80% and the accuracy rate can reach 86.30%, which is better than other models. Experiments 6 and 7 show that the exhibition of BERT is superior to that of word2vec, so that the F1 values and accuracy of other RNN models represented by Experiments 1 to 5 are significantly ahead of those of Experiment 7. From Experiment 1 to Experiment 8, the transformer encoder has better feature extraction ability than RNN. In addition, Experiments 7 and 8 show that the multilevel information interaction of the model in this paper does improve the effect of short-text matching, mainly reflected in the improvement of F1 value and accuracy. The reason why LSTM model achieves better matching effect is that it can solve the problem of polysemy by using the Bert model for text vectorization. At the same time, the transformer encoder has better feature extraction ability. The multilevel information interaction makes the two texts get rich interactive information, which has a better effect on short-text matching.

#### 4.4.2. Scoring Effect of Ideological and Political Texts

After training and integrating semantic integrity analysis model and short-text similarity calculation model, subjective item can be scored. We think that if the difference between automatic scoring and manual scoring is no more than 10% of the total score (10 points), the automatic scoring is correct; otherwise, it is an error. We use greedy strategy and global optimal strategy to score the 50 reserved “standard answer -student answer” pairs. The accuracy results of the two strategies compared with the real manual scoring are shown in Figure 5.

Randomly select a sample of subjective test set in the final examination of ideological and political course for freshmen in a university and load the students' answers and reference answers in the subjective item scoring system. The test paper numbers of students' answers are 01, 02,…, 49, and 50, respectively.

From the selected samples, it can be clearly seen that generally ideal scoring results have been accomplished partially. There are a few distinctions in the scoring consequences of certain examples. This error may be composed of the following two parts. One is the text segmentation model proposed in this paper. There are few improper word segmentations in word segmentation. The other situation may be that the subjective items are evaluated manually, which may be caused by personal subjective opinions. On the whole, the ideological and political education text scoring model based on improved transformer has achieved relatively ideal results in practical application.

On the basis of all the previous improvements, as we expected, the global optimal strategy has a good scoring effect and is obviously better than the greedy strategy. The greedy strategy only focuses on the current maximum value, and the selected scores are often quite different. However, the global optimal strategy starts from the whole, and the selected scores are more evenly distributed, which is in line with the situation that teachers grade students' answers according to the score points in real life.

## 5. Conclusion

Under the background of intelligent education, this paper presents an automatic scoring algorithm for subjective questions in ideological and political lessons. Aiming at the problem that the accuracy of similarity calculation of long text is not high, a short-text similarity calculation model based on transformer is constructed, which is used to calculate the similarity between each score point in the standard answer and each clause in the student's answer, so as to achieve better scoring effect. The test results show that the transformer encoder has better feature extraction ability, multi-level information interaction enables the two texts to obtain rich interactive information, and the matching effect of short text is better improved. In the practical application of ideological and political teaching, the ideal effect has been achieved. However, for the training of the model, we did not take data with different sample sizes, and the training time of the model was not tested. Further work will be carried out around this.

## Figures and Tables

**Figure 1:** The process of automatic scoring algorithm of subjective item in politics ideological and political course.

**Figure 2:** Structure of the transformer encoder.

**Figure 3:** Model convergence.

**Figure 4:** Comparison of different models.

**Figure 5:** Comparison of scoring effects of different scoring strategies.

**Table 1:** Experimental parameter setting.

Parameter	Value
Encoder layers	2
Number of attention heads	8
Hidden layer dimension	768
Dropout	0.10
Model optimizer	Adam
Maximum sequence length	25
Batch_size	512

## Data Availability

The data included in this study are available upon request by contact with the corresponding author.
